# An Inexact Penalty Decomposition Method for Sparse Optimization

**DOI:** 10.1155/2021/9943519

**Published:** 2021-07-14

**Authors:** Zhengshan Dong, Geng Lin, Niandong Chen

**Affiliations:** ^1^College of Mathematics and Data Science, Minjiang University, Fuzhou 350108, China; ^2^New Huadu Business School of Minjiang University, Minjiang University, Fuzhou 350108, China

## Abstract

The penalty decomposition method is an effective and versatile method for sparse optimization and has been successfully applied to solve compressed sensing, sparse logistic regression, sparse inverse covariance selection, low rank minimization, image restoration, and so on. With increase in the penalty parameters, a sequence of penalty subproblems required being solved by the penalty decomposition method may be time consuming. In this paper, an acceleration of the penalty decomposition method is proposed for the sparse optimization problem. For each penalty parameter, this method just finds some inexact solutions to those subproblems. Computational experiments on a number of test instances demonstrate the effectiveness and efficiency of the proposed method in accurately generating sparse and redundant representations of one-dimensional random signals.

## 1. Introduction

In this paper, we consider solving the following sparse optimization problem by an inexact penalty decomposition (iPD) method:

(1) $$\begin{array}{c} \underset{x\in X}{\min}\;l\left(x\right)+\lambda {\left\|x\right\|}_{0},\\ \text{s.t.}g\left(x\right)\leq 0,h\left(x\right)=0, \end{array}$$

where *λ* ≥ 0 controls the sparsity of the solution, *𝒳* ⊂ *ℝ*^*n*^ is a closed convex set in the *n*-dimensional Euclidean space *ℝ*^*n*^, *l* : *ℝ*^*n*^⟶*ℝ*, *g*(*x*) : *ℝ*^*n*^⟶*ℝ*^*p*^ are continuously differentiable convex functions, *h* : *ℝ*^*n*^⟶*ℝ*^*m*^ is an affine function, and ‖*x*‖_0_ denotes the number of nonzero components of *x*.

Sparse optimization is to solve some problems whose solutions are sparse or compressed. And it has attracted considerable attention in the past ten years since its broad applications, such as signal (image) processing [1–3], linear regression [4], inverse problem [5], model selection [6], and machine learning [6, 7]. In those applications, most information of interest has or can be coded by much low dimension though its own dimension is high.

However, problem (1) is NP hard even though for some simple special cases [8]. Even so, many methods have been proposed for some special cases of problem (1). These methods can be classified into four categories: (1) greedy methods: matching pursuit [9, 10] and greedy coordinate descent [11]; (2) *l*_1_-norm relaxation methods: gradient projection [12, 13], iterative shrinkage-thresholding [5, 14], iterative reweighted method [15], alternating direction method [16], and homotopy method [17–20]; (3) *l*_*p*_-norm (0 < *p* < 1) relaxation methods [1, 2, 21]; and (4) *l*_0_-norm based methods, e.g., penalty decomposition method [22], block decomposition method [23], iterative hard thresholding method [22, 24–29], and so on. In this paper, we mainly discuss the PD method.

The PD method was proposed for solving the general *l*_0_-norm minimization problem (1) by Lu and Zhang in [22]. And it had been successfully applied to solve compressed sensing [22], sparse logistic regression [22], sparse inverse covariance selection [22], low rank minimization [30], image restoration [3] problems, and so on. Moreover, the PD method is theoretically sound. Lu et al. stated that any accumulation point of the sequence generated by the PD method satisfies the first-order optimality conditions of problem (1) when the Robinson condition holds. Hence, the PD method is an effective and versatile method for sparse optimization. However, since the PD method found exact solutions of subproblems for each penalty parameter, it may be time consuming in practice.

In this paper, an inexact penalty decomposition (iPD) method is proposed for the sparse optimization problem (1). The iPD method just finds some inexact solutions to those subproblems for each penalty parameter. In more detail, for the first convex subproblem, the iPD method just takes one gradient step and then goes to solve the second nonconvex subproblem. The second subproblem can be solved by the iterative hard thresholding method [26]. After the two steps, the penalty parameter is updated. Computational experiments on a number of random instances demonstrate the effectiveness of the proposed method in accurately generating sparse and redundant representations of one-dimensional random signals.

The rest of this paper is organized as follows.  Section 2 is the preliminary, in which some notations and the basic method are described.  Section 3 presents the iPD method. Computational experiments are presented in Section 4, and conclusions are drawn in Section 5.

## 2. Preliminaries

### 2.1. Notations

In this subsection, some notations are presented to simplify presentation. The transpose of a vector *x* ∈ *ℝ*^*n*^ is denoted by *x*^*T*^. If without special statement, all norms used are the Euclidean norm, denoted by ‖·‖_2_. *𝒫*_*𝒳*_(·) denotes projection on a set *𝒳*. Given a vector *x* ∈ *ℝ*^*n*^, the nonnegative part of *x* is denoted by *x*^+^, i.e., *x*^+^=max(*x*, 0). The index of nonzero components of a vector *x* is denoted by *S*(*x*)={*i* :  *x*_*i*_ ≠ 0} (called support set) and *S*_*k*_ : =*S*(*x*^*k*^). The size of *S*(*x*) is denoted as *s*=|*S*(*x*)|.

Now, let us consider problem (1). It is easy to verify that problem (1) is equivalent to the following problem:

(2) $$\begin{array}{c} \underset{x,y\in X}{\min}\;l\left(x\right)+\lambda {\left\|y\right\|}_{0},\\ \text{s.t.}g\left(x\right)\leq 0,h\left(x\right)=0,\;x=y. \end{array}$$

And the relative penalty function of problem (2) is defined as

(3) $$\begin{array}{c} p_{\rho }\left(x,y\right)=l\left(x\right)+\lambda {\left\|y\right\|}_{0}+\frac{\rho }{2}\left({\left\|{\left[g\left(x\right)\right]}^{+}\right\|}_{2}^{2}+{\left\|h\left(x\right)\right\|}_{2}^{2}+{\left\|x-y\right\|}_{2}^{2}\right), \end{array}$$

where *ρ* > 0 is the penalty parameter.

For simplicity, we also denote

(4) $$\begin{array}{c} F_{\rho }\left(x\right)=l\left(x\right)+\lambda {\left\|x\right\|}_{0}+\frac{\rho }{2}\left({\left\|{\left[g\left(x\right)\right]}^{+}\right\|}_{2}^{2}+{\left\|h\left(x\right)\right\|}_{2}^{2}\right),\\ f\left(x\right)=\frac{1}{2}\left({\left\|{\left[g\left(x\right)\right]}^{+}\right\|}_{2}^{2}+{\left\|h\left(x\right)\right\|}_{2}^{2}\right),\\ q_{\rho }\left(x,y\right)=l\left(x\right)+\frac{\rho }{2}\left({\left\|{\left[g\left(x\right)\right]}^{+}\right\|}_{2}^{2}+{\left\|h\left(x\right)\right\|}_{2}^{2}+{\left\|x-y\right\|}_{2}^{2}\right). \end{array}$$

### 2.2. The PD Method

In this subsection, we show the PD method proposed in [22]. First, the outline of the PD method is as presented in Algorithm 1. Then, we explain why the PD method is time consuming by a random example.

**Remark 1 .**

(i) The termination condition in Step 8 of Algorithm 1 is used to establish the global convergence of the PD method. In practice, the termination criterion is based on the relative change of the sequence {(*x*^*k*,*i*^, *y*^*k*,*i*^)} such as the sequence satisfying

(5) $$\begin{array}{c} \max\left\{\frac{{\left\|x^{k,i}-x^{k,i-1}\right\|}_{\infty }}{\max\left({\left\|x^{k,i}\right\|}_{\infty },1\right)},\frac{{\left\|y^{k,i}-y^{k,i-1}\right\|}_{\infty }}{\max\left({\left\|y^{k,i}\right\|}_{\infty },1\right)}\right\}\leq \epsilon_{I}, \end{array}$$

for some *ϵ*_*I*_ > 0. In addition, the PD method terminates the outer iterations when

(6) $$\begin{array}{c} {\left\|x^{k}-y^{k}\right\|}_{\infty }\leq \epsilon_{O}, \end{array}$$

holds for some *ϵ*_*O*_ > 0.

(ii) The second subproblem, i.e., in Step 6 of Algorithm 1,

(7) $$\begin{array}{c} y^{k,i+1}\in \underset{y}{\arg\min}\lambda {\left\|y\right\|}_{0}+\frac{\rho_{k}}{2}{\left\|y-x^{k,i+1}\right\|}_{2}^{2}, \end{array}$$

has a closed-form solution [26].

(8) $$\begin{array}{c} y_{j}^{k,i+1}=\left\{\begin{array}{cc} x_{j}^{k,i+1}, & \text{if }\left|x_{j}^{k,i+1}\right|>\sqrt{\frac{2\lambda }{\rho_{k}}},\\ 0, & \text{otherwise}, \end{array}\right. \end{array}$$

where [·]_*j*_ denotes the *j*-th entry of a vector, *j* ∈ {1,2,…, *n*}.

In Step 5 of Algorithm 1, minimizing the function *p*_*ρ*_*k*__(*x*, *y*^*k*^) with respect to *x* is a convex problem. There exist many efficient methods for this purpose if *𝒳* is simple. However, for each penalty parameter, the PD method solves the penalty subproblems a few times until some termination conditions are reached, which is time consuming.

Consider a special case—compressed sensing [31]. One important task of compressed sensing is to find the sparsest solution to the underdetermined linear system, which is formulated as

(9) $$\begin{array}{c} \underset{x}{\min}\;{\left\|x\right\|}_{0},\\ \text{s.t.}Ax=b, \end{array}$$

where *A* ∈ *ℝ*^*m*×*n*^ is the sensing matrix and *b* ∈ *ℝ*^*m*^ is the observation data. For this special problem, *f*(*x*)=(1/2)‖*Ax* − *b*‖_2_^2^ and *F*_*ρ*_(*x*)=‖*x*‖_0_+(*ρ*/2)‖*Ax* − *b*‖_2_^2^. The value of *f*(*x*) is called data fidelity, and it can measure the feasibility of a solution *x*. *F*_*ρ*_(*x*) is the penalty function of problem (9).

**Example 1 .**

We generate a sparse vector ${\bar{x}}^{*}$ with length *n*=5000 and *s*=100 nonzero components. These components independently follow the standard Gaussian distribution, and their locations are assigned randomly to ${\bar{x}}^{*}$. Then, we create a Gaussian random matrix *A* with size 1000 × 5000, and let $b=A{\bar{x}}^{*}$. Then, we solve this instance by the PD method package, and the process data are presented as Figure 1.

Figure 1 shows that the value of *f*(*x*) decreases slowly. It decreases steep just at the first few steps for each penalty parameter. There are many almost null steps during the process. And the value of the penalty function *F*_*ρ*_(*x*) increases too much when updating the penalty parameter. Hence, we can just take one or a few iterations for each penalty parameter to save some time.  In Section 3, we will improve the PD method by the above observations.

## 3. The Proposed Method

In this section, we describe the process of the iPD method. From the outline of Algorithm 1, we find that, for each penalty parameter *ρ*_*k*_, the block coordinate descent method needs to alternately solve two minimization subproblems many times, and an example in Section 2 shows that there are many almost null step for each penalty parameter. Hence, the original PD method may be time consuming if convergence speed of the block coordinate descent is slow.

Motivated by the analysis in Section 2 and the above demonstration, we accelerate the PD method by alteratively solving the two penalty subproblems once a time after updating the penalty parameter. For solving the first penalty subproblem, a gradient step is taken, and its step-length is searched by the backtracking line search method.

Now, we present the outline of the accelerated penalty decomposition method as follows.

**Remark 2 .**

A practical termination criterion in Step 11 of Algorithm 2 can be

(10) $$\begin{array}{c} \frac{{\left\|x^{k}-y^{k}\right\|}_{\infty }}{\max\left({\left\|x^{k}\right\|}_{\infty },1\right)}\leq \text{tol}, \end{array}$$

for some tol > 0.

**Theorem 1 .**

If the gradient of the function *p*_*ρ*_*k*__(*x*, *y*^*k*^) with respect to *x* is Lipschitz continuous (its Lipschitz constant is denoted as *L*_*p*_), then the line search between Steps 3–6 can be terminated in a finite number of iterations.

**Proof**

Since *p*_*ρ*_*k*__(*x*^*k*+1^, *y*^*k*^) satisfies

(11) $$\begin{array}{c} p_{\rho_{k}}\left(x^{k+1},y^{k}\right)\leq p_{\rho_{k}}\left(y^{k},y^{k}\right)+\nabla_{x}p_{\rho_{k}}{\left(y^{k},y^{k}\right)}^{T}\left(x^{k+1}-y^{k}\right)+\frac{L_{p}}{2}{\left\|x^{k+1}-y^{k}\right\|}_{2}^{2}, \end{array}$$

it together with *x*^*k*+1^=*y*^*k*^ − (∇_*x*_*p*_*ρ*_*k*__(*y*^*k*^, *y*^*k*^)/*L*_*k*_) implies that

(12) $$\begin{array}{c} p_{\rho_{k}}\left(x^{k+1},y^{k}\right)\leq p_{\rho_{k}}\left(x,y^{k}\right)-\left(L_{k}-\frac{L_{p}}{2}\right){\left\|x^{k+1}-x^{k}\right\|}_{2}^{2}. \end{array}$$

Then, if *L*_*k*_ ≥ ((*L*_*p*_+*η*)/2),

(13) $$\begin{array}{c} p_{\rho_{k}}\left(x^{k+1},y^{k}\right)+\frac{\eta }{2}{\left\|x^{k+1}-y^{k}\right\|}_{2}^{2}\leq p_{\rho_{k}}\left(y^{k},y^{k}\right), \end{array}$$

holds, which means that the while loop in Algorithm 2 terminates if *L*_*k*_ ≥ ((*L*_*p*_+*η*)/2). Let ${\bar{L}}_{k}$ be the final value of *L*_*k*_ after the while loop. Then, $\left({\bar{L}}_{k}/\gamma_{\text{inc}}\right)\leq \left(\left(L_{p}+\eta \right)/2\right)$ holds, i.e., ${\bar{L}}_{k}\leq \left(\gamma_{\text{inc}}\left(L_{p}+\eta \right)/2\right)$. Let ${\hat{n}}_{k}$ be the number of iterations in the while loop at the *k*-th iteration. Then, one can get that

(14) $$\begin{array}{c} L_{\min}\gamma_{\text{inc}}^{{\hat{n}}_{k}-1}\leq L_{k}^{0}\gamma_{\text{inc}}^{{\hat{n}}_{k}-1}\leq {\bar{L}}_{k}\leq \frac{\gamma_{\text{inc}}\left(L_{p}+\eta \right)}{2}, \end{array}$$

where *L*_*k*_^0^ is the initial value of *L*_*k*_ in the line search. Therefore,

(15) $$\begin{array}{c} {\hat{n}}_{k}\leq N≔\left\lceil \frac{\log\left(L_{p}+\eta \right)-\log\left(2L_{\min}\right)}{\log\left(\gamma \right)}+2\right\rceil . \end{array}$$

## 4. Experiments

In this section, we implement the proposed accelerated PD method to solve the compressed sensing problem. To verify the efficiency of PD empirically, a large number of computational experiments are performed on one-dimensional random signals. We mainly compare the performance of our improved PD method with that of the original PD method [22]. All experiments were performed on a personal computer with an Intel(R) Core(TM)i7-7700HQ CPU (2.80 GHz) and 8 GB memory, using a MATLAB toolbox (version R2018b).

We compare the performance of the compared methods by the CPU time (in seconds) required, the size of the support set of the reconstructed data $\hat{x}$, and the mean squared error (MSE) with respect to ${\bar{x}}^{*}$, which is defined as

(16) $$\begin{array}{c} \text{MSE}=\frac{1}{n}\left\|\hat{x}-{\bar{x}}^{*}\right\|, \end{array}$$

and the data fidelity of $A\hat{x}-y$ is defined as

(17) $$\begin{array}{c} \text{DF}=\frac{1}{2}{\left\|A\hat{x}-y\right\|}^{2}, \end{array}$$

and NS as the number of successfully recovered instances. We say a signal $\hat{x}$ is successfully recovered if the positions of the nonzero components of $\hat{x}$ are the same as ${\bar{x}}^{*}$ and the corresponding MSE value is less than 10^−4^.

### 4.1. Data Generation and Parameter Setting

Each instance is generated randomly with size (*m*, *n*, *s*), where *m* × *n* is the dimension of matrix *A* and *s* is the sparsity level, such as *m*=1000, *n*=5000, and *s*=100. The elements of matrix *A* follow the Gaussian distribution. The vector ${\bar{x}}^{*}$ is generated with the same distribution at *s* randomly chosen coordinates. Finally, the vector *b* is generated by $b=A{\bar{x}}^{*}$.

Unless otherwise stated, all parameters in the PD method are set as default, and parameters in the IPD package are set as in Table 1.

### 4.2. Compare with the Original PD Method

Firstly, we compare the iteration process of the iPD method with that of the PD method on a random instance. All parameters are set as before, and the problem size is *m*=1000, *n*=5000,  and *s*=100.  Figure 2 describes the data fidelity and the penalty function value over the iteration process. From Figure 2(a), we find that the iPD method does not have many null steps, and the values of data fidelity generated by the iPD method decrease much fast than those of the original PD method. Furthermore, the iPD method just requires about 150 steps while the original PD method requires about 400 steps. And the running time of the iPD method is about 7 seconds, which is less than half of the time required by the original PD method. Moreover, the penalty function value generated by the iPD method is much stable than that by the original PD method.

In the second experiment, we compare the accelerated PD method with its original PD method at different sampling numbers. We fix the dimension *m*=5000 and the sparsity level *s*=100. For each sampling number *m*, 100 instances are generated, and the averaged performance of the two methods is presented in Figure 3.

From Figure 3(a), we see that the accelerated PD method requires not more than 10 seconds while the original PD method requires much more time. And the time required by the accelerated PD method is stable at different sampling numbers.  Figure 3(b) shows that the recovered rate by the accelerated PD method is higher than that by the original PD method when *m* is bigger than 600. When the sampling number is bigger than 700, the accelerated PD method can recover all signals successfully. We find that the MSE value and the DF value generated by the accelerated PD method are lower than those generated by the original PD method. The averaged number of nonzero components also shows that the accelerated PD method performs better.

In the next experiment, we compare the accelerated PD method with its original version for solving the compressed sensing problem with different sparsity levels *s*. All parameters are set as the same value as those stated before. The averaged computational results on 100 instances are presented in Table 2.

From Table 2, we find that the PD method not works well when the sparsity level is greater than 150, especially when it is greater than 200. However, the sparsity level recovered by the iPD method can reach 200. When the two methods can recover sparse signals, the iPD method just needs about one third of the time required by the PD method. Moreover, the recovered rate of the iPD method is higher than that of the original PD method. From MSE and DF value, we see that the signals recovered by the iPD method are more exact than those recovered by the PD method. When *s*=100, there is one instance not recovered exactly by the iPD method since there exist several very small components and one of them is not recovered.

## 5. Conclusions

In this paper, we have proposed an acceleration of the penalty decomposition for the sparse approximation problem. The proposed method does not solve the penalty subproblems exactly and alternately solve penalty subproblems once a time after updating penalty parameters. We show that this method enhances the performance of the penalty decomposition method by computational experiments on a number of random instances for solving the compressed sensing problem. The experiments demonstrate that the proposed method indeed improves the original PD method since it recovers better solutions with less running time.

## Figures and Tables

**Figure 1:** Iteration process of penalty decomposition for solving compressed sensing with size *m*=1000, *n*=5000,  and *s*=100: (a) data fidelity at each iteration; (b) penalty function value at each iteration.

**Figure 2:** Iteration process of the compared methods for solving compressed sensing with size *m*=1000, *n*=5000,  and *s*=100: (a) data fidelity at each iteration; (b) penalty function value at each iteration.

**Figure 3:** Averaged results of the penalty decomposition methods for the compressed sensing problem with different sampling numbers on 100 instances: (a) CPU time over sampling number; (b) recovered rate over sampling number; (c) MSE over sampling number; (d) data fidelity over sampling number; (e) number of nonzero components over sampling number.

**Algorithm 1:** : The PD method [22].

**Algorithm 2:** : The inexact PD method.

**Table 1:** Parameter settings in the acceleration of the PD method.

Parameter	Value
*x*_0_	0
*ρ*	*ρ*_0_=10, *ρ*_*k*+1_=min(1.1*ρ*_*k*_, 10^15^)
tol	10^−6^
*η*	1
*L*	*L*_0_=0.1max(‖*A*_*j*_‖_2_^2^) *γ*_inc_=2, *γ*_dec_=3

**Table 2:** Averaged results on 100 instances with size *m*=1000 and *n*=5000 for each sparsity level *s*

Algorithm	*s*	Time (s)	NNZ	MSE	DF	NS
PD	50	18.2	50	5.62 × 10^−9^	5.95 × 10^−7^	100
	100	21.69	99.95	1.06 × 10^−8^	2.61 × 10^−6^	95
	150	26.36	149.88	2.50 × 10^−8^	3.50 × 10^−5^	89
	200	76.38	297.65	6.72 × 10^−5^	8.19 × 10^−2^	73
	250	102.54	1225.21	1.22 × 10^−3^	3.53 × 10^−1^	0
	270	105.18	1283.92	1.58 × 10^−3^	1.93 × 10^−1^	0

iPD	50	6.72	50	3.22 × 10^−9^	1.77 × 10^−7^	100
	100	8.56	99.99	5.20 × 10^−9^	3.62 × 10^−7^	99
	150	9.78	150	7.31 × 10^−9^	5.85 × 10^−7^	100
	200	10.32	200	9.32 × 10^−9^	7.66 × 10^−7^	100
	250	11.75	656.87	5.50 × 10^−5^	1.03 × 10^−6^	30
	270	12.75	1235.9	3.67 × 10^−4^	9.72 × 10^−7^	1

## Data Availability

The data used to support the findings of this study are included within the article.
